RETRACTED

# Combination of alpha-synuclein immunotherapy with anti-inflammatory treatment in a transgenic mouse model of multiple system atrophy

**DOI:** 10.1186/s40478-016-0409-1

**Published:** 2017-01-05

**Authors:** Elvira Valera, Brian Spencer, Jerel A. Fields, Ivy Trinh, Anthony Adame, Michael Mante, Edward Rockenstein, Paula Desplats, Eliezer Masliah

**Affiliations:** 1 Department of Neurosciences, University of California, 9500 Gilman Drive, La Jolla, San Diego, CA 92093-0624 USA; 2 Department of Pathology, University of California, 9500 Gilman Drive, La Jolla, San Diego, CA 92093-0624 USA

**Keywords:** Multiple system atrophy, Alpha-synuclein, Immunotherapy, Single-chain antibody, Lenalidomide, Neuroinflammation

## Abstract

Multiple system atrophy (MSA) is a fatal neurodegenerative disorder characterized by the pathological accumulation of alpha-synuclein (α-syn) in oligodendrocytes. Therapeutic efforts to stop or delay the progression of MSA have yielded suboptimal results in clinical trials, and there are no efficient treatments currently available for MSA patients. We hypothesize that combining therapies targeting different aspects of the disease may lead to better clinical outcomes. To test this hypothesis, we combined the use of a single-chain antibody targeting α-syn modified for improved central nervous system penetration (CD5-D5) with an unconventional anti-inflammatory treatment (lenalidomide) in the myelin basic protein (MBP)-α-syn transgenic mouse model of MSA. While the use of either CD5-D5 or lenalidomide alone had positive effects on neuroinflammation and/or α-syn accumulation in this mouse model of MSA, the combination of both approaches yielded better results than each single treatment. The combined treatment reduced astrogliosis, microgliosis, soluble and aggregated α-syn levels, and partially improved behavioral deficits in MBP-α-syn transgenic mice. These effects were associated with an activation of the Akt signaling pathway, which may mediate cytoprotective effects downstream tumor necrosis factor alpha (TNFα). These results suggest that a strategic combination of treatments may improve the therapeutic outcome in trials for MSA and related neurodegenerative disorders.

**Electronic supplementary material:**

The online version of this article (doi:10.1186/s40478-016-0409-1) contains supplementary material, which is available to authorized users.

## Introduction

Multiple system atrophy (MSA) is a rapidly progressive and fatal neurodegenerative disease characterized by parkinsonism, dysautonomia [5, 56], and accumulation of the protein alpha-synuclein (α-syn) within oligodendroglial cells in the form of glial cytoplasmic inclusions [16, 19] leading to neuroinflammation, demyelination and neurodegeneration [15, 25, 43, 47, 50, 57]. The lack of response to levodopa and the extensive accumulation of α-syn within oligodendrocytes differentiates MSA from other synucleinopathies [6, 55]. MSA is an orphan neurodegenerative disorder with no effective disease-modifying treatment, and recent clinical trials of MSA therapies have failed to meet primary endpoints [7, 23, 30, 35]. These negative results were probably associated with the late diagnosis of this disorder, and treatments being initiated when α-syn accumulation and neuroinflammation are already widespread.

RETRACTED

Regarding potential therapies for MSA, some anti-inflammatory treatments have shown promise at the preclinical level [42, 46, 50], and therapies aimed at reducing neuroinflammation are currently being tested in clinical trials (Clinical trial identifiers NCT02388295, NCT02315027). We have recently explored the use of antidepressants [50] and immunomodulatory drugs [48] as therapeutics in animal models of synucleinopathy. We observed that the antidepressants fluoxetine, olanzapine and amitriptyline not only ameliorate neuroinflammation, but also reduce the accumulation of α-syn in the Myelin Basic Protein (MBP)-α-syn transgenic (tg) mouse model of MSA [50]. Moreover, another unconventional anti-inflammatory, the anticancer drug and immunomodulatory compound lenalidomide, was able to effectively reduce microgliosis and the expression of pro-inflammatory cytokines in an animal model of Parkinson’s disease (PD) [48], a disorder also characterized by the accumulation of α-syn. Lenalidomide is a small thalidomide derivative with anti-angiogenic and immunomodulatory activity, that has shown therapeutic effects in multiple myeloma [3, 31, 45] and in animal models of Amyotrophic lateral sclerosis [28, 44]. Its mechanisms of action are multiple, primarily involving T cell co-stimulation [14, 18, 59], increased NK cell proliferation and function [18, 59], and inhibition of the production of TNFα [13, 31, 59] and other proinflammatory cytokines [4]. We selected lenalidomide for this study because preliminary reports showed that this compound is also effective at reducing neuroinflammation in the tg mouse model used in this study ([49], and unpublished data). Moreover, these results suggest that the repurposing of FDA-approved compounds may speed up the search for an effective therapy for MSA.

Immunotherapy has also shown promise for treating neurodegenerative disorders; moreover, active immunotherapeutic approaches are under consideration for the treatment of MSA patients (Clinical trial identifier NCT02270489). Regarding passive immunotherapy, we have recently developed a single-chain antibody against α-syn that is conjugated to the LDL receptor-binding domain of apolipoprotein B (ApoB), which allows the antibody to readily cross the blood-brain barrier [40]. Systemic expression of this antibody effectively reduced neuronal α-syn accumulation in a tg mouse model of synucleinopathy [40]. Moreover, the modified single-chain antibody showed enhanced brain penetration and was imported into neuronal cells through the endosomal sorting complex required for transport (ESCRT) pathway, leading to lysosomal degradation of α-syn aggregates. Further analysis showed that this antibody was also effective at ameliorating neurodegenerative pathology, neuroinflammation and behavioral deficits observed in the mouse model of synucleinopathy [40].

RETRACTED

These exciting results reported by others and ourselves led us to hypothesize that combining FDA-approved immunomodulatory compounds with our successful immunotherapeutic strategy might be beneficial for the treatment of synucleinopathies. The rationale is that combining treatments targeting different aspects of the disease (i.e. neuroinflammation plusα-syn accumulation) may enhance the beneficial effects of single therapies. Therefore, the goal of the current study is to test in vivo the feasibility and efficacy of a combination of α-syn immunotherapy and anti-inflammatory treatment for MSA and related disorders.

## Materials and methods

### Animal model and treatments

Mice expressing human α-syn under the control of the MBP promoter (MBP-α-syn tg, line 1) were generated as previously described [38]. MBP-α-syn tg mice develop progressive accumulation of α-syn inclusions in oligodendrocytes along the axonal tracts in the brainstem, basal ganglia, cerebellum, corpus callosum, and neocortex, leading to neurodegeneration in the neocortex and to loss of dopaminergic fibers in the basal ganglia. Non-tg and MBP-α-syn tg mice (*n* = 12–14 per condition and genotype) were administered by intraperitoneal injection of a lentiviral construct expressing the single-chain antibody CD5-D5 linked to ApoB sequence (LV-CD5-D5-ApoB), or LV-control (100 μl/mouse, 1 × 10^9^ transducing units). As previously described [8, 40], the anti-oligomeric α-syn single-chain antibody (D5) cDNA was amplified by PCR and cloned into the third-generation self-inactivating lentivirus vector plasmid [41] with the CMV promoter driving expression. D5 is linked to the secretory signal from the human CD5 gene [17] and to the LDL receptor-binding domain from apolipoprotein B (apoB) [40]. The construct also includes a V5 tag for immunodetection (Additional file 1).

One week after injection, mice were treated with lenalidomide (100 mg/kg) or vehicle (0.5% methocellulose) daily for 4 weeks (*n* = 6–7 per condition and genotype). Fresh vehicle or lenalidomide preparations were administered via gavage in a 5 ml/kg volume. All mice were between 10 and 11 months of age by the end of the study. All experiments were carried out in accordance with the guidelines set by the NIH regarding the care and use of animals for experimental procedures. All animal procedures were approved by the UCSD Institutional Animal Care and Use Committee.

RETRACTED

### Behavioral analyses

The behavioral assessment of the animals was performed using open field 1 week before endpoint. As previously described [34], animals were evaluated for 10 min for three consecutive days, given a 2-day dishabituation period, followed by a fourth and final trial. Context-dependent learning was collected using a Kinder SmartFrame Cage Rack Station activity monitor system (Kinder Scientific), in 3-dimentional space using a 7x15 beam configuration. Data collection began when an animal was placed in the test chamber. Total activity and rearing (i.e. standing on rear limbs) were calculated as total beam breaks in 10 min, and thigmotaxis was calculated as the percentage of time spent in the periphery.

### Immunohistochemistry

Mice were sacrificed under anesthesia following NIH guidelines for the humane treatment of animals, and brains were removed. The right hemibrain was fixed by immersion in 4% paraformaldehyde in PBS pH 7.4 and serially sectioned at 40 μm with a Vibratome apparatus (Leica) for subsequent analysis. The left hemibrain was stored at −80 °C for biochemical analysis, and further processed for either quantitative real-time polymerase chain reaction (qPCR) or protein analysis.

Vibratome sections were immunolabeled overnight with antibodies against α-syn (Sigma, 1:250), Glial fibrillary acidic protein (GFAP) (Millipore, 1:500), Iba1 (Wako, 1:2000) or MAP2 (Millipore, 1:500), followed by incubation with species-appropriate secondary antibodies (Vector Laboratories). Sections were reacted with 3,3’-diaminobenzidine (Vector Laboratories) and imaged on an Olympus BX41 microscope. A minimum of 100 cells were counted per animal, and cell counts are expressed as the average number of positive cells per field (230 μm x 184 μm). Quantification of GFAP and Iba1 staining was performed by obtaining optical density measurements using the Image Quant 1.43 program (NIH) and corrected against background signal levels.

### Immunoblotting and ELISA assay

Protein homogenates were prepared from the mouse posterior hemibrain. Briefly, frozen samples were sonicated in homogenization buffer (HEPES 1 mM, benzamidine 5 mM, 2-mercaptoethanol 2 mM, EDTA 3 mM, MgSO_4_ 0.5 mM, NaN_3_ 0.05%, protease inhibitor cocktail set III 1:100, phosphatase inhibitor cocktail set II 1:100) and ultracentrifuged at 100,000 rpm for 1 h to obtain cytosolic (soluble) and particulate (insoluble, membrane-bound) fractions. 20 μg of protein from the cytosolic or particulate fractions were loaded onto 4–12% Bis-Tris SDS-PAGE gels (Invitrogen) and transferred onto Immobilon membranes. After overnight incubation with antibodies against total α-syn (Millipore), phospho- and total p38 (Abcam, Cell Signaling Technologies), phospho- and total Akt (Cell Signaling Technologies), phospho- and total ERK1/2 (Cell Signaling Technologies), tumor necrosis α (TNFα) (Santa Cruz), MBP (BioRad), CNPase (Sigma) or Olig2 (IBL International), membranes were incubated in HRP-linked secondary antibody (American Qualex), reacted with ECL Western blotting substrate (Perkin Elmer) and developed in a VersaDoc gel-imaging system (BioRad). An antibody against β-actin was used as loading control. Immunoblotting images were analyzed using Quantity One software (BioRad).

RETRACTED

Levels of human α-syn were determined in the cytosolic fraction of mouse brain homogenates by an ELISA assay (Invitrogen) according to the manufacturer’s protocol. 2.5 μg of protein were used per animal per reaction, and concentration of α-syn was calculated by extrapolating from a human α-syn standard curve.

### RNA isolation and real time PCR

Total RNA was extracted from the mouse anterior hemibrain using a Qiagen RNeasy kit and following the instructions of the manufacturer. 0.5 μg of RNA per sample were used for reverse transcription to cDNA using a High capacity cDNA reverse transcription kit (Applied Biosystems). qPCR was performed using TaqMan Fast Advanced Master Mix and the appropriate TaqMan primers (Life Technologies). qPCR reactions were run in an StepOnePlus Real-Time PCR system and ΔΔCt calculations [36] were made using StepOne software (Applied Biosystems).

### Statistical analysis

Values are expressed as average ± standard error of the mean (SEM). To determine the statistical significance we used one-way analysis of variance (ANOVA) with Dunnett post-hoc test when comparing to the control condition. Additional comparisons were done using Tukey post hoc test. The differences were considered to be significant if p values were less than 0.05.

## Results

### Combined treatment with lenalidomide and CD5-D5 ameliorates neuroinflammation in the MBP-α-syn transgenic mouse model of MSA

The pathological accumulation of α-syn within oligodendrocytes observed in MSA brains, and reproduced in tg mouse models of MSA, is typically associated with an increase in neuroinflammation markers [52]. The astrogliosis and microgliosis present in MSA brains may have deleterious effects such as potentiating neurodegeneration and α-syn accumulation. Therefore, reducing neuroinflammation may represent a promising therapeutic goal in MSA patients. We have recently explored the use of anti-inflammatory molecules in MSA models [50], and have analyzed the effects of lenalidomide in a mouse model of PD [48]. Moreover, passive immunization of α-syn tg mice with the single-chain anti-α-syn antibody CD5-D5 also reduced neuroinflammation [40].

RETRACTED

In the current study we explored the neuroprotective effects of the combined treatment of lenalidomide and CD5-D5 in the MBP-α-syn tg mouse model of MSA. Immunohistochemistry results showed that the combined treatment reduced astrogliosis in the corpus callosum and striatum, as measured by GFAP immunostaining (Fig. 1). Specifically, the optical density of the GFAP signal was increased by 60 and 70% in the corpus callosum and striatum, respectively, of the tg mice compared to non-tg controls; lenalidomide and CD5-D5 treatment returned GFAP signal to that of control mice (Fig. 1b, c). This effect seems to be mostly due to the anti-inflammatory effect of lenalidomide, as it can be deduced by comparing to the lenalidomide-only treatment. Moreover, the optical density of the Iba1 signal was increased by 30 and 100% in the corpus callosum and striatum, respectively, of the tg mice compared to non-tg controls; lenalidomide and CD5-D5 treatment returned Iba1 signal to that of control mice (Fig. 1b, c). Both lenalidomide treatment and immunotherapy had a similar inhibitory effect on microgliosis, and the combined treatment showed no synergistic effect. A more detailed analysis of microglial morphology revealed that striatal Iba1-positive cells from MBP-α-syn tg mice show increased ramification, and that both single and combined treatments reduced the number of branches per cell (Additional file 2), mirroring optical density results. Moreover, treatment with lenalidomide and/or CD5-D5 increased microglial cell soma diameter in the striatum of tg animals [54], suggesting a shift in microglial polarization towards phagocytic state as a consequence of the immunotherapy [2, 20]. Finally, additional analysis of neuronal dendritic arborization using MAP2 immunostaining revealed a significant increase in striatal dendritic density with lenalidomide or CD5-D5 treatment, and a surge in the number of dendritic ramifications with both single and combined treatments (Additional file 3).

**Fig. 1:** Combined treatment reduces astrogliosis and microgliosis in MBP-α-syn transgenic mice. **a**-**c** Representative images of GFAP immunostaining and optical density quantification in neocortex (**a**), corpus callosum (**b**) and striatum (**c**) of non-tg and MBP-α-syn tg mice treated with LV-control or LV-CD5-D5-ApoB, and vehicle or lenalidomide. **d**-**f** Representative images of Iba1 immunostaining and optical density quantification in neocortex (**d**), corpus callosum (**e**) and striatum (**f**) of non-tg and MBP-α-syn tg mice treated with LV-control or LV-CD5-D5-ApoB, and vehicle or lenalidomide. Results are presented as average ± SEM. * *p* < 0.05, ** *p* < 0.01 and *** *p* < 0.001 when comparing vehicle/LV-control-treated non-tg mice to vehicle/LV-control-treated tg mice. # *p* < 0.05, ## *p* < 0.01 and ### *p* < 0.001 when comparing vehicle/LV-control-treated tg mice to single or multi-treated tg mice. Scale bar = 25 μm

It has been postulated that reducing neuroinflammation may prevent the downstream toxic effects of α-syn. Our results suggest that lenalidomide is effective at reducing neuroinflammation in a tg mouse model of MSA, and that its combination with an anti-α-syn approach does not have adverse inflammatory effects in mice.

RETRACTED

### Combined treatment with lenalidomide and CD5-D5 reduces α-syn accumulation in the MBP-α-syn transgenic mouse model of MSA

Immunotherapy against α-syn has been effective at reducing α-syn accumulation in different models of synucleinopathy, and it is currently under investigation for its efficacy in human patients. We measured the accumulation of α-syn by immunohistochemistry, immunoblot and ELISA in the brain of MBP-α-syn tg mice treated with lenalidomide and/or CD5-D5 (Fig. 2). The combined treatment of lenalidomide and CD5-D5 significantly reduced the accumulation of α-syn in all brain areas analyzed by 75–80% (Fig. 2a-c). This effect was 2–3 times stronger than treatment with CD5-D5 alone, suggesting that combination with lenalidomide may potentiate or trigger additional clearance mechanisms. This reduction not only affected α-syn aggregates (insoluble α-syn), as the combined treatment also reduced soluble α-syn measured by immunoblot and ELISA (Fig. 2d, f). These results further support the use of this type of combined treatment, as it improves the results obtained by single therapies, which are by themselves less efficient.

**Fig. 2:** Combined treatment reduces α-syn accumulation in MBP-α-syn transgenic mice. **a**-**c** Representative images of α-syn immunostaining and cell counts in neocortex (**a**), corpus callosum (**b**) and striatum (**c**) of non-tg and MBP-α-syn tg mice treated with LV-control or LV-CD5-D5-ApoB, and vehicle or lenalidomide. **d** Immunoblot and densitometric analysis of α-syn in the soluble fraction of protein extracts from non-tg and MBP-α-syn tg mice treated with LV-control or LV-CD5-D5-ApoB, and vehicle or lenalidomide. Significant results of three mice per group are shown. **e** Immunoblot and densitometric analysis of α-syn in the insoluble fraction of protein extracts from non-tg and MBP-α-syn tg mice treated with LV-control or LV-CD5-D5-ApoB, and vehicle or lenalidomide. Significant results of three mice per group are shown. **f** ELISA analysis of human α-syn levels in the soluble fraction of protein extracts from non-tg and MBP-α-syn tg mice treated with LV-control or LV-CD5-D5-ApoB, and vehicle or lenalidomide. Results are presented as average ± SEM. *** *p* < 0.001 when comparing vehicle/LV-control-treated non-tg mice to vehicle/LV-control-treated tg mice. # *p* < 0.05, ## *p* < 0.01 and ### *p* < 0.001 when comparing vehicle/LV-control-treated tg mice to single or multi-treated tg mice. Scale bar = 25 μm

It can be suggested that either or both of treatments may be altering the number of mature oligodendrocytes instead of reducing α-syn accumulation. Preliminary tests with lenalidomide in the MBP-α-syn tg mouse model revealed that this compound did not alter the number of mature oligodendrocytes as measured by p25α immunostaining (data not shown). MBP and CNPase protein levels were not significantly reduced in MBP-α-syn tg animals (Additional file 4), consistent with the fact that the tg mouse line used in this study shows less myelin pathology than higher α-syn expressor lines [38]. Interestingly, the levels of early oligodendroglial precursor cell (OPC) marker Olig2 showed a trend to the increase in tg animals (Additional file 4), in line with previous studies reporting an increase in OPC numbers in this mouse model, and a blockage in OPC differentiation [9, 26]. Neither of the treatments had a significant effect on oligodendrocyte marker levels (Additional file 4), suggesting that the changes observed in α-syn accumulation were likely due to the clearance of intracellular aggregates.

RETRACTED

### Combined treatment with lenalidomide and CD5-D5 modulates TNFα expression and activates Akt signaling in the MBP-α-syn transgenic mouse model of MSA

To determine the effect of combining lenalidomide and immunotherapy againstα-syn on the inflammatory response, we analyzed the expression of the cytokine TNFα in the brain of MBP-α-syn tg mice treated with lenalidomide and/or CD5-D5 (Fig. 3a, b). Release of TNFα by microglia has been traditionally associated to neuroinflammation, and it mediates pro-inflammatory cascades associated to cytotoxicity [12, 32]. Lenalidomide was originally developed as an anti-TNFα molecule, and has been shown to reduce both TNFα mRNA and protein levels [31, 59]. We observed that levels of soluble TNFα were reduced approximately 40% in the mouse brain with lenalidomide treatment (Fig. 3a, b). A trend for the increase of soluble TNFα in the brain of tg animals treated with either CD5-D5 or combined treatment was also observed (Fig. 3a, b), indicating that antibody treatment counteracts the TNFα-reducing effects of lenalidomide in this mouse model. Levels of membrane-bound (insoluble) TNFα were significantly elevated by 50% in MBP-α-syn tg mice, and were not altered by any of the treatments (Fig. 3a, b). These results suggest that even though antibody treatment appears to be neutralizing the anti-TNFα effects of lenalidomide, the neuropathological analysis showing reduced neuroinflammation with the combined treatment (Fig. 1) indicates that this modulation of TNFα expression does not translate into reduced anti-inflammatory effects. Furthermore, it is possible that a mild activation of microglia elicited by immunotherapy may be behind these changes.

**Fig. 3:** Combined treatment modulates TNFα expression and Akt signaling in MBP-α-syn transgenic mice. **a** Immunoblot analysis of the levels of soluble and insoluble (membrane-bound) TNFα in non-tg and MBP-α-syn tg mice treated with LV-control or LV-CD5-D5-ApoB, and vehicle or lenalidomide. Significant results of three mice per group are shown. **b** Densitometric analysis of the levels of soluble and insoluble (membrane-bound) TNFα in non-tg and MBP-α-syn tg mice treated with LV-control or LV-CD5-D5-ApoB, and vehicle or lenalidomide. **c** Immunoblot and densitometric analysis of phospho- and total Akt and phospho- and total ERK1/2 in the soluble fraction of protein extracts from non-tg and MBP-α-syn tg mice treated with LV-control or LV-CD5-D5-ApoB, and vehicle or lenalidomide. Significant results of three mice per group are shown. **d** Densitometric analysis of the levels of the phospho- and total Akt, and phospho- and total ERK1/2 immunoreactive bands, normalized by actin levels and expressed as phospho/total ratio. Results are presented as average ± SEM. ** *p* < 0.01 when comparing vehicle/LV-control-treated non-tg mice to vehicle/LV-control-treated tg mice. ## *p* < 0.01 when comparing vehicle/LV-control-treated non-tg mice to multi-treated non-tg mice, or vehicle/LV-control-treated tg mice to single or multi-treated tg mice

TNFα activates pro-inflammatory signals, usually associated to p38, JNK and ERK1/2 (MAPKs) downstream pathways [53]. However, in certain cases TNFα can also activate cytoprotective signaling, that may be associated to Akt activation [11]. Immunoblot analysis confirmed a significant reduction in phosphorylated (activated) Akt in MBP-α-syn tg animals compared with non-tg littermates (Fig. 3c, d). Both lenalidomide and CD5-D5 significantly increased phospho-Akt in tg animals, with the combined treatment achieving the higher Akt activation (Fig. 3c, d). However, all of the treatments showed a trend for a reduction in ERK1/2 phosphorylation (Fig. 3c, d). Levels of phosphorylated p38 were not increased by any of the treatments (not shown). These results, together with the neuropathology data, suggest that the activation of Akt signaling and the reduction of ERK1/2 signaling may coordinately achieve a cytoprotective effect in this tg model. Moreover, these results further confirm the anti-inflammatory potential of the combined treatment at the molecular level.

RETRACTED

### Combined treatment with lenalidomide and CD5-D5 modulates behavioral changes in the MBP-α-syn transgenic mouse model of MSA

To determine if lenalidomide and CD5-D5 reverses behavioral deficits, animals were also analyzed using the open field monitoring system (Fig. 4). While MBP-α-syn tg animals showed no changes in hyperactivity phenotype when compared to non-tg littermates, we did observe a significant decrease in rearing and a trend to reduction of total activity with the combined treatment (Fig. 4a, b), suggesting that the treatment may have hyperactivity-reducing effects. Thigmotaxis, a measure of anxiety, was not significantly altered with any of the treatments (Fig. 4c). The behavioral modification achieved with the treatment seemed to be mostly due to CD5-D5 treatment. More research is needed in models with stronger hyperactivity phenotype to further determine the full extent of behavioral improvements that could be induced by the combined treatment.

**Fig. 4:** Combined treatment modulates behavioral changes in MBP-α-syn transgenic mice. Non-tg and tg animals treated with LV-control or LV-CD5-D5-ApoB, and vehicle or lenalidomide were analyzed in the open field test. **a** Total activity, measured as total beam breaks. **b** Rearing, measured as total beam breaks. **c** Thigmotaxis, measured as the percentage of time spent in the periphery. Results are presented as average ± SEM. # *p* < 0.05 when comparing vehicle/LV-control-treated tg mice to single or multi-treated tg mice

## Discussion

Effective treatments for orphan neurodegenerative disorders like MSA are sorely needed. Unfortunately for MSA patients, several promising therapeutic compounds recently failed in clinical trials, and identifying novel interventions is challenging the traditional process of drug discovery. In the current study we investigate the therapeutic efficacy of combining an unconventional anti-inflammatory therapy (lenalidomide) with an α-syn-reducing immunotherapeutic approach (CD5-D5 single-chain antibody) in a novel tg mouse model for MSA pathogenesis. Interestingly, we observed that the combined treatment achieves better results than each treatment alone in a tg mouse model of MSA. Together, lenalidomide and CD5-D5 significantly reduced astrogliosis, microgliosis, and soluble and insoluble α-syn accumulation (results are summarized in Fig. 5). The combined treatment increased the activation of the Akt signaling pathway, that has been previously associated with cytoprotective effects in the brain. Finally, the treatment also ameliorated some behavioral measurements in this tg mouse model. Similar to successful treatment regiments for diseases such as HIV and cancer, these results indicate that combining two or more compatible therapies might have increased therapeutic potential when compared to using single therapies for the treatment of neurodegenerative disorders.

RETRACTED

**Fig. 5:** Proposed mechanism of action of the combined treatment with lenalidomide and CD5-D5. In the MBP-α-syn transgenic mouse model of MSA, oligodendrocytes produce high levels of α-syn, leading to the pro-inflammatory activation of microglia and astroglia. The diagram shows the mechanism of action of lenalidomide and LV-CD5-D5-ApoB in the MBP-α-syn transgenic mouse brain. The combined treatment with lenalidomide (Len) and LV-CD5-D5-ApoB (D5) reduces oligodendroglial α-syn accumulation, modulates astroglial activation, regulates the expression of cytokines, and activates the cytoprotective Akt signaling. Immunotherapy with LV-CD5-D5-ApoB may also target extracellular α-syn, promoting its uptake by microglial cells and reducing its incorporation into astroglial cells. The combined treatment also increases the expression of TNFα mRNA, which could be linked to the observed inhibition of ERK1/2 in favor of Akt signaling

For the first time, we show that combining lenalidomide and an anti-α-syn antibody with enhanced penetration to the CNS achieves better results than treatment with either one alone in a tg mouse model of MSA. This is the case of the reduction observed in the number of α-syn-positive cells in all brain areas analyzed, and the reduction in rearing in MBP-α-syn tg mice treated with the combination of both therapies. In other cases, the effect of the combined treatment could be attributed to one of the treatments (Fig. 5). Interestingly, we did not observe that the combined treatment worsened any of the parameters analyzed, and it always achieved equal or better outcomes than either of the single treatments.

Lenalidomide and CD5-D5 modulate both shared and treatment-specific pathways in glial cells. While lenalidomide is a potent anti-inflammatory [28, 48], CD5-D5 seems to act through stimulation of brain cells to uptake and clear α-syn [40], achieving a reduction in neuroinflammation. Alternatively, CD5-D5 may reduce neuroinflammation through an indirect mechanism downstream of the activation of α-syn clearance mechanisms. Interestingly, we observed greater reduction in α-syn levels with the combined treatment than with each treatment alone, supporting the idea of combined treatments as a better alternative for MSA and other synucleinopathies. Interestingly, we also observed a reduction in α-syn accumulation with lenalidomide treatment in the MBP-α-syn tg animals, while we previously failed to observe such reduction in the mThy1-α-syn tg mouse model of PD [48]. This discrepancy may be due to the intrinsic differences between these two models of synucleinopathy. The mThy1-α-syn tg mice express human α-syn in neurons [33] while MBP-α-syn tg express it in oligodendrocytes (glia) [38], which may react differently to lenalidomide treatment. It is also possible that the reduction in α-syn accumulation achieved by lenalidomide is an indirect effect of its modulatory effect on the phagocytic activity of microglial cells [22, 48]. Finally, we cannot rule out the possibility of lenalidomide altering α-syn propagation, as we have observed before with other anti-inflammatory treatments such as the antidepressant fluoxetine [50].

RETRACTED

It is important to consider that lenalidomide and other anti-inflammatory compounds modulate the immune system, and this effect should be taken into consideration when simultaneously modulating microglial responses with an anti-inflammatory and stimulating microglia with an immunotherapeutic treatment. To prevent an interaction between the treatments that may neutralize some of the desired effects, we administered immunotherapy 1 week before lenalidomide treatment. Moreover, the dual effects of lenalidomide and CD5-D5 in microglial activation may explain the signaling results observed. Lenalidomide was initially developed as an anti-TNFα molecule that effectively reduces mRNA and protein levels of TNFα in cancer models [31]. Lenalidomide alone reduced the levels of soluble TNFαmeasured in total RNA from whole brain extracts, however the combined treatment failed to induce a reduction in the levels of soluble TNFα. Such disparities highlight the complex regulation of cytokine expression in the brain, and in particular that achieved by combining drugs that may have complementary effects on immune cells. We hypothesize that the effect observed in TNFα levels could be due to a mild activation of microglia by the immunotherapy to stimulate α-syn clearance, an effect that has been previously observed in other immunotherapy studies [24, 27, 37]. Importantly, the detected changes in TNFα levels were not associated with increased astrogliosis or microgliosis, as demonstrated in Fig. 1.

RETRACTED

TNFα has been traditionally associated with pro-inflammatory changes in the diseased brain [1, 39], however several studies have suggested that TNFα may also play an anti-inflammatory role [10, 21]. Interaction of TNFα with TNFR1 has been associated with activation of p38, JNK and ERK1/2 leading to inflammation and cytotoxicity [51], while binding to TNFR2 is associated with the activation of signaling cascades that promote cytoprotection [51]. Furthermore, TNFR2 stimulation in microglia regulates the expression of genes involved in immune processes, including molecules with anti-inflammatory and neuroprotective function [51]. While activation of Akt signaling can be pro-inflammatory in some cases, the activation of the Akt signaling pathway may improve cell survival depending on the receptor upstream Akt activation [29, 58]. Further research will be needed to elucidate how the combined treatment, but not each treatment separately, is able to activate cytoprotective pathways.

## Conclusions

In conclusion, our results show that the combination of an anti-inflammatory treatment with an α-syn-reducing treatment has better disease-modifying effects than each treatment alone in an animal model of MSA. These results open the door for the design of more complex clinical trials in which a carefully planned combination of therapies can complement each other to target multiple aspects of the pathology. However, more research will be necessary to investigate how molecular pathways weave together to potentially achieve synergism without eliciting unwanted deleterious effects in patients with neurodegenerative disorders.

## Additional files

Additional file 1: V5 immunostaining confirms the expression of the single-chain antibody CD5-D5-ApoB. (A) Representative images of V5 immunostaining (LV-CD5-D5-ApoB tag) in the neocortex of non-tg and MBP-α-syn tg mice treated with LV-control or LV-CD5-D5-ApoB, and vehicle or lenalidomide. (B) Cell counts of V5-positive cells in in the neocortex of non-tg and MBP-α-syn tg mice treated with LV-control or LV-CD5-D5-ApoB, and vehicle or lenalidomide. (TIF 1365 kb)
Additional file 2: Morphological analysis of striatal microglia by Iba1 immunostaining. (A) Representative high-magnification images of Iba1 immunostaining in the striatum of non-tg and MBP-α-syn tg mice treated with LV-control or LV-CD5-D5-ApoB, and vehicle or lenalidomide. Inverted images were used for quantification purposes. (B) Quantification of microglial ramification as measured by the number of branches per cell. (C) Microglial soma size as measured by the maximum soma diameter. A minimum of 20 cells were quantified per animal. Results are presented as average ± SEM. * *p* < 0.05, and *** *p* < 0.001 when comparing vehicle/LV-control-treated non-tg mice to vehicle/LV-control-treated tg mice. ## *p* < 0.01 and ### *p* < 0.001 when comparing vehicle/LV-control-treated tg mice to single or multi-treated tg mice. Scale bar = 20 μm. (TIF 1825 kb)
Additional file 3: Analysis of striatal dendritic arborization by MAP2 immunostaining. (A) Representative high-magnification images of striatal MAP2 immunostaining in the striatum of non-tg and MBP-α-syn tg mice treated with LV-control or LV-CD5-D5-ApoB, and vehicle or lenalidomide. Inverted images were used for quantification purposes. (B) Quantification of dendritic density as measured by the percentage of MAP2 positive area. (C) Quantification of dendritic arborization as measured by the number of MAP2 positive branches per μm^2^. Results are presented as average ± SEM. ** *p* < 0.01, and *** *p* < 0.001 when comparing vehicle/LV-control-treated non-tg mice to vehicle/LV-control-treated tg mice. #*p* < 0.05, ## *p* < 0.01 and ### *p* < 0.001 when comparing vehicle/LV-control-treated tg mice to single or multi-treated tg mice. (TIF 1704 kb)
Additional file 4: Immunoblot analysis of oligodendroglial and myelination markers. (A) Immunoblot analysis of the levels of MBP, CNPase and Olig2 in non-tg and MBP-α-syn tg mice treated with LV-control or LV-CD5-D5-ApoB, and vehicle or lenalidomide. Significant results of three mice per group are shown. (B) Densitometric analysis of the levels of MBP, CNPase and Olig2 in non-tg and MBP-α-syn tg mice treated with LV-control or LV-CD5-D5-ApoB, and vehicle or lenalidomide. Results are presented as average ± SEM. (TIF 1161 kb)

RETRACTED

## Abbreviations

ANOVA: Analysis of variance
ApoB: Apolipoprotein B
CNS: Central nervous system
ESCRT: Endosomal sorting complex required for transport
GFAP: Glial fibrillary acidic protein
LV: Lentivirus
MBP: Myelin basic protein
MSA: Multiple system atrophy
OPC: Oligodendroglial precursor cell
PD: Parkinson’s disease
TNFR: Tumor necrosis factor α receptor
TNFα: Tumor necrosis factor α
α-syn: α-synuclein
